The article "Predictive Value of HPV E6/E7 mRNA Detection on the Outcome of Cervical LSIL" was retracted in 2023. Reasons: signs of a paper mill; suspected computer-generated content; unreliable results or conclusions; concerns about the data.

# Predictive Value of HPV E6/E7 mRNA Detection on the Outcome of Cervical LSIL

**DOI:** 10.1155/2022/8747919

**Published:** 2022-08-08

**Authors:** Limei Cao, Ping He, Jun Yang, Xin Long, Yanqiu Chen, Li Yan, Deping Zhou

**Affiliations:** Department of Obstetrics and Gynecology, Women and Children's Hospital of Chongqing Medical University, Chongqing 400000, China

## Abstract

*Objective*. To assess the predictive worth of HPV E6/E7 mRNA detection in the outcome of the cervical low-grade squamous intraepithelial lesion (LSIL). From September 2017 to early September 2019, patients screened for high-risk HPV positive or abnormal cervical liquid-based cytology were retrospectively analyzed and diagnosed with LSIL by cervical biopsy were recruited. The independent influencing factors of the regression of LSIL lesions after follow-up were analyzed, and the outcome of LSIL was calculated. The results of the initial colposcopy in this study were CIN I, CIN II/P16-negative, CIN II/P16-positive, and CIN III. At the time of re-examination, LSIL patients had three outcomes: regression, persistence, and progression. In the two follow-ups, 330 patients were finally included, including 276 CIN I patients (group A) and 54 CIN II/P16-negative patients (group B). The positive rates of HPV E6/E7 mRNA in each group were 66.67% and 70.37% for A and B, respectively. The total positive rate of E6/E7 mRNA was 67.27%, and there was no significant difference between the two groups (*P* > 0.05). After 1 year follow-up, whether HPV E6/E7 mRNA regressed or was negative was associated with the outcome of LSIL-related lesions (*P* < 0.05). The regression or negative rate of HPV E6/E7 mRNA was 1.57 times higher than the progression rate of HPV E6/E7 mRNA-positive diagnosis of LSIL lesions. Univariate logistic regression analysis showed that age at first sexual intercourse, HPV E6/E7 mRNA results, and lesion type were statistically significant (*P* < 0.05). Whether HPV E6/E7 mRNA was negative (OR = 2.420, *P*=0.001) and age at first sexual intercourse ≥20 years (OR = 0.420, *P*=0.002) were independent influencing factors associated with LSIL regression. Multivariate logistic analysis showed that age of first sexual intercourse ≥20 years (OR = 0.420, *P*=0.002) and HPV E6/E7 mRNA-negative (OR = 2.420, *P*=0.001) were independent factors associated with LSIL. HPV E6/E7 mRNA detection can be used for predicting the outcome of LSIL and has a good application value.

## 1. Introduction

Cervical cancer is a malignant tumor that occurs frequently in the female reproductive system. Research shows that the global incidence of cervical cancer is as high as 500,000 new cases every year [1]. In China, 2nd highest incidence of cervical cancer among women aged 15–44, after breast cancer, and the mortality rate ranks third. The occurrence of cervical cancer is inextricably linked with human papillomavirus (HPV), and HPV can be discovered in 99.7% of cervical cancers [2]. Persistent high-risk HPV infection is the main reason for cervical cancer and the vast majority of cervical precancerous lesions [3]. Cervical intraepithelial neoplasia (CIN) is precancerous lesion closely related to cervical invasive carcinoma. Early detection of CIN through cervical cancer screening, timely treatment of CIN, timely diagnosis, and reasonable treatment and follow-up management are effective measures to prevent cervical cancer [4]. The vast majority of LSILs in CIN resolve spontaneously, and only a few persistently progress to cervical cancer [5]. At present, the commonly used screening methods such as vaginal and cervical smears, Pap tests, and HPV DNA detection cannot identify persistent HPV infection [6] and cannot predict the biological behavior of CIN, that is, cannot judge its clinical characteristics. Outcomes result in the current overtreatment or undertreatment of cervical precancerous lesions. At present, HPV E6/E7 mRNA detection has been approved for clinical application. Previous studies have reported that in cervical tissue with low-grade lesions, the possibility of malignant transformation of cervical lesions in HPV E6/E7 mRNA-negative patients is very low, while in cervical tissue with high-grade lesions, the accuracy and negative predictive value of HPV E6/E7 mRNA were higher than those of HPV E6/E7 DNA [7]. However, whether it has value in predicting the prognosis and outcome of CIN lesions has not yet been concluded. Therefore, this research intends to evaluate the use value of HPV E6/E7 mRNA detection in projecting the result of cervical LSIL, which is reported as follows.

## 2. Materials and Methods

### 2.1. General Information

The research subjects were screened from sexually active women who were referred from other hospitals or other departments in our hospital to our hospital's cervical disease specialist because of high-risk HPV-positive or abnormal cervical liquid-based cytology results from September 2017 to September 2019. The clinical data of the selected patients were collected, and the patient's age, pregnancy, number of sexual partners, age at first sex, menstruation, marriage and childbearing history, contraception history, disease history, tumor family history, and educational background were recorded. Inclusion criteria were as follows: age 18–45 years old; sufficient colposcopy results; colposcopy found lesions and site biopsy and pathological diagnosis of LSIL (including CIN I and CIN II and P16 negative); no previous history of cervical cancer and CIN; nonpregnant period; and patient informed consent. Exclusion criteria were as follows: vaccinated against HPV vaccine; previous precancerous lesions of the vulva and vagina; precancerous lesions or malignant tumors in other parts; autoimmune diseases or diseases that require immunosuppressive agents, such as systemic Lupus erythematosus, glomerulonephritis, and those who received physical therapy or drug therapy during the follow-up period. This study was approved by the medical ethics committee of our hospital, and the subjects participated voluntarily and signed the informed consent.

### 2.2. Methods

1. After the patients were enrolled, pathologists detected HPV E6/E7 mRNA (Aptima, Hologic, USA) in accordance with the kit instructions. The cervical exfoliated cell specimens were obtained by brush and placed in the preservation solution and then transferred to the pathology department for HPV E6/E7 mRNA detection. The test results were kept in the pathology department, and statistics were carried out after the follow-up. The method uses capture hybridization to detect 14 high-risk subtypes (HPV 16, 18, 31, 33, 35, 39, 45, 51, 52, 56, 58, 59, 66, and 68), and for HPV16, 18/45 perform type testing. All tests were expressed as the ratio of the sample measurement value/reference value; with a ratio ≥1.0, the result was “positive;” and with a ratio <1.0, the result was “negative.”
2. After the medical staff collected the cervical epithelial cells of the enrolled patients, they used the liquid-based ultra-thin cytology technology (TCT) to prepare and read the films. Diagnostic criteria [8]: pathological diagnosis using cervical intraepithelial neoplasia, three-level classification (CIN I, CIN II, and CIN III), and two classifications (cervical LSIL and HSIL), parallel two classification methods. P16 immunohistochemical staining was performed for CIN II lesions, and the positive ones were classified as HSIL, and the negative ones were classified as LSIL. During the 1-year follow-up in this study, neither doctors nor patients were aware of the HPV E6/E7 mRNA test results.

### 2.3. Observation and Evaluation Indicators

1. To analyze the relationship and predictive value of different HPV E6/E7 mRNA expressions and lesion outcomes
2. Binary logistic regression was used to analyze the independent influencing factors related to LSIL regression statistical methods

### 2.4. Statistical Methods

SPSS 23.0 version was applied for data analysis, count data were expressed as rate (%), the chi-square test was applied for comparison between groups, and the rank sum test was applied for independent group rank count data. A binary logistic regression model was used to analyze the independent influencing factors related to the prognosis of LSIL lesions, and the 95% confidence interval (CI) of the OR value was calculated. *P* < 0.05 was supposed statistically important.

## 3. Results

### 3.1. Analysis of the Relationship between HPV E6/E7 mRNA and Lesion Outcome

The results of the initial colposcopy histological examination were CIN I, CIN II/P16-negative, CIN II/P16-positive, and CIN III. The re-examination results showed that the lesions of LSIL patients regressed, persisted, and progressed (Figure 1).

### 3.2. Colposcopy Results

A total of 330 patients were eligible for inclusion and completed two follow-up visits, including 276 patients with CIN I (group A) and 54 patients with negative CIN II/P16 (group B). The overall positive rate was 67.27% (222/330), the positive rate of group A was 66.67%, and the positive rate of group B was 70.37%. There was no statistical difference between the two groups (*P*=0.596). The composition ratio of other 11 types was not statistically different (*P*=0.428), as given in Table 1 and Figure 2.

### 3.3. The Relationship and Predictive Value of HPV E6/E7 mRNA Detection Results and Lesion Outcome

Between the two visits, 36 patients were upgraded to HSIL (10.9%), 92 patients continued to LSIL (27.9%), and 202 patients had disease resolution (61.2%). The relationship and predictive value of different HPV E6/E7 mRNA expressions and lesion outcomes were analyzed. It was found that whether HPV E6/E7 mRNA was negative after a 1-year follow-up, and the type of lesion was associated with the outcome of LSIL lesions (*P*=0.012). Among the 36 patients with progressive LSIL lesions, 22 had HPV E6/E7 mRNA regressed or negative, 14 had HPV E6/E7 mRNA persistently positive, and HPV E6/E7 mRNA regressed or negative rates were HPV E6/E7 mRNA-positive diagnosis of LSIL lesions 1.57 times the progression rate. Among the 92 patients with persistent LSIL lesions, 52 had HPV E6/E7 mRNA regressed or negative, and 40 were persistently positive. HPV E6/E7 mRNA regression or negative rate was 1.3 times the progression rate of HPV E6/E7 mRNA-positive diagnosis of LSIL lesions. Of the 202 patients with regressed LSIL lesions, 148 had regressed or negative HPV E6/E7 mRNA and 54 had persistently positive HPV E6/E7 mRNA, as given in Table 2.

### 3.4. Univariate Analysis Affecting the Outcome of LSIL

Lesion outcome was divided into regressed and nonregressed (persistent and progressive) as a binary outcome. Univariate logistic regression analysis was performed. The results showed that the age at first sexual intercourse, HPV E6/E7 mRNA results and lesion type were statistically significant (*P* < 0.05), as given in Table 3.

### 3.5. Binary Logistic Regression Analysis and Multivariate Analysis Related to the Outcome of LSIL

The factors with statistical significance in the univariate analysis were included in the multivariate analysis, and the distribution is given in Table 4. The analysis results showed that the age of first sexual intercourse ≥20 years of age (OR = 0.420, *P*=0.002) and whether HPV E6/E7 mRNA was negative (OR = 2.420, *P*=0.001) were independent factors associated with LSIL, as given in Table 5.

## 4. Discussion

According to previous reports, LSIL is mostly caused by HPV sexual infection, most of which can be cleared by the body's immune system. It can be seen that LSIL has a high natural negative rate. However, due to the preventive examination of vaginal and cervical smears, Pap test and HPV DNA detection, and other screening methods, the prognosis of LSIL patients cannot be well predicted, and there are many clinical overtreatment and treatment of LSIL patients. The phenomenon of frequent biopsies [9]. Therefore, in order to avoid overtreatment and frequent poor detection in LSIL patients, it is of great significance to find new detection methods to predict the outcome of LSIL.

Previous studies have reported that the oncogenic proteins encoded by HR-HPV E6/E7 genes are generally in a dormant state, and persistent infection with HPV virus can activate the expression of HPV E6 gene, resulting in the degradation of the tumor suppressor gene p53, while the HPV E7 gene is in a dormant state. Combine with the tumor suppressor gene Rb to degrade it, eventually leading to the occurrence of malignant tumors. Both E6 and E7 are important factors leading to CIN [10–12]. HR-HPV E6/E7 mRNA test is a promising noninvasive biomarker; compared with the HPV DNA test, HPV mRNA test and DNA test are in good agreement, in the detection of high-grade cervical lesions (CIN II+). It has similar sensitivity and higher specificity, suggesting that it can not only detect HPV infection but also predict changes in cervical lesions [13, 14]. Ratnam et al. [15] claimed that detection of HPV E6/E7 oncogene expression may be more predictive of cervical cancer risk than detection of HPV DNA. Liu et al. [16] believed that the positive expression of E6/E7 mRNA has a certain predictive value for the follow-up evaluation of CIN II+ in women with negative colposcopy. The results of Wang et al. [17] and others showed that the positive expression of HPV E6/E7 mRNA has a good predictive value for HSIL+. Ho et al. [18] reported that the expression level of HPV E6/E7 mRNA was highly correlated with the severity of cervical lesions. The results of this study showed that after a 1-year follow-up, the regression rate of LSIL lesions was about 60% and the progression rate was about 10%. Whether the HPV E6/E7 mRNA turned negative after one year and the type of lesions were related to the outcome of LSIL lesions. There was no difference in the positive rate of HPV E6/E7 mRNA and the proportion of HPV type 16 and type 18/45 in the CIN I and CIN II/P16-negative subgroups of this group of patients. Therefore, patients with CIN I and CIN II/P16-negative patients can be combined as LSIL for management.

When E6/E7 mRNA is detected, it means that the HPV oncogene has been integrated into infected cells and may gradually develop into malignant lesions. Therefore, some scholars speculate that HPV E6/E7 mRNA may be related to the prognosis of lesions. Liu [19] and others followed up 32 CIN I-II patients and found that patients with both E6 and E7 mRNAs had an increased risk of disease progression compared with other patients. A meta-analysis showed that compared with negative patients, HPV E6/E7 mRNA-positive patients had a higher risk of developing HSIL in the next 2 years [20]. Wang et al. [21] followed up CIN I patients with normal or mildly abnormal cytology for two years and found that the incidence of lesion progression in the HPV E6/E7 mRNA positive group was significantly higher than that in the 12, 18, and 24 months of follow-up. Negative group, the higher the expression of E6/E7 mRNA, the greater the possibility of CIN I progression.

In this research, the outcome of cervical LSIL patients was analyzed from different HPV E6/E7 mRNA results; it turns out that HPV E6/E7 mRNA regressed or negative patients was better than that of HPV E6/E7 mRNA-positive patients. Therefore, clinical attention should be paid to patients with HPV E6/E7 mRNA-positive. In this research, the independent influencing factors related to LSIL regression were analyzed by multivariate regression analysis. The results displayed that whether HPV E6/E7 mRNA was positive at the time of enrollment was not associated with the prognosis of LSIL and whether HPV E6/E7 mRNA was negative during a 1-year follow-up and the age of first sexual life ≥ 20 is related to the regression of LSIL lesions, suggesting that the focus should be on the age of first sexual life <20 years old, and the follow-up of such patients should be strengthened to detect the HPV E6/E7 mRNA.

This research is a small sample analysis, and the conclusions have great limitations. Some enrolled patients were referred from other hospitals or interdepartmental referrals in the hospital. The HPV detection methods used initially before enrollment were different, so it was impossible to compare the worth of HPV E6/E7 mRNA in the prognosis of LSIL lesions compared with other HPV detection methods. Subsequent studies can use the comparative study design of HPV DNA detection and simultaneous detection of E6/E7 mRNA detection to contrast the advantages and disadvantages of the two.

In general, the detection of HPV E6/E7 mRNA can predict the outcome of LSIL and has a good application value. One-year follow-up of LSIL patients if HPV E6/E7 mRNA changes from positive to negative or continues to be negative; it is predicted that LSIL may subside. If HPV E6/E7 mRNA remains positive, clinical intervention should be actively performed.

## Figures and Tables

**Figure 1:** Analysis of the relationship between HPV E6/E7 mRNA and lesion outcome.

**Figure 2:** The positive rate of colposcopy.

**Table 1:** Colposcopy results.

Colposcopy results	Total	Group A (*n* = 276)	Group B(*n* = 54)	*P*
Negative	108	92 (33.33%)	16 (29.63%)	0.596
Positive	222	184 (66.67%)	38 (70.37%)	
Type 16	66	55 (19.93%)	11 (20.37%)	0.428
Type 18/45	37	28 (10.14%)	9 (16.67%)	
Other type 11	119	101 (36.59%)	18 (33.33%)	

**Table 2:** The relationship and predictive value of HPV E6/E7 mRNA detection results and lesion outcome.

HPV E6/E7 mRNA results	Lesion outcome			*P*
	Remission (*n* = 202)	Persistent (*n* = 92)	Progression (*n* = 36)	
HPV E6/E7 mRNA				0.943
Positive	136 (67.33%)	61 (66.30%)	25 (69.44%)	
Negative	66 (32.67%)	31 (33.70%)	11 (30.56%)	

HPV E6/E7 mRNA				0.012
Regression or negative	148 (73.27%)	52 (56.52%)	22 (61.11%)	
Persistent positive	54 (26.73%)	40 (43.48%)	14 (38.89%)	

Type of disease				0.089
CIN I	145 (71.78%)	55 (59.78%)	22 (61.11%)	
CIN II/P16-negative	57 (28.22%)	37 (40.22%)	14 (38.89%)	

**Table 3:** Univariate analysis affecting the outcome of LSIL.

Basic features	Remission (*n* = 202)	Nonremission (*n* = 128)	*χ* ^2^	*P*
Age (years old)			0.077	0.782
<35	82 (40.59%)	50 (39.06%)		
≥35	120 (59.41%)	78 (60.94%)		
Pregnancy (time)			0.355	0.551
<2	125 (61.88%)	75 (58.59%)		
≥2	77 (38.12%)	53 (41.41%)		
Number of partners			0.974	0.324
<3	143 (70.79%)	84 (65.63%)		
≥3	59 (29.21%)	44 (34.37%)		
Age of first sexual intercourse (years old)			5.800	0.016
<20	52 (25.74%)	49 (38.28%)		
≥20	150 (74.26%)	79 (61.72%)		
Condoms for contraception			3.068	0.080
Yes	72 (35.64%)	58 (45.31%)		
No	130 (64.36%)	70 (54.69%)		
Education level			2.271	0.132
College and above	78 (38.61%)	39 (30.47%)		
Below college	124 (61.39%)	89 (69.53%)		
HPV E6/E7 mRNA			0.001	0.979
Positive	136 (67.33%)	86 (67.19%)		
Negative	66 (32.67%)	42 (32.81%)		
HPV E6/E7 mRNA			8.500	0.004
Regression or negative	148 (73.27%)	74 (57.81%)		
Persistent positive	54 (26.73%)	54 (42.19%)		
Type of disease			4.810	0.028
CIN I	145 (71.78%)	77 (60.16%)		
CIN II/P16-negative	57 (28.22%)	51 (39.84%)		

**Table 4:** Argument assignment table.

Independent variable	Assignment method
Age of first sexual intercourse	<20 = 0; ≥20 = 1
HPV E6/E7 mRNA	Regression or negative = 0; persistent positive = 1
Type of disease	CIN I = 0; CIN II/P16-negative = 1

**Table 5:** Binary logistic regression analysis and multivariate analysis related to LSIL outcomes.

Variable	*β*	Standard error	Wald *χ*^*2*^	*P*	OR	95% CI
Age of first sexual intercourse	−0.771	0.336	4.484	0.002	0.420	0.243–0.727
HPV E6/E7 mRNA	0.175	0.067	6.806	0.001	2.420	1.419–4.127
Type of disease	0.951	0.540	3.101	0.031	1.790	1.053–3.042

## Data Availability

The data used to support the findings of this study are available from the corresponding author upon request.
